# Differential Prognostic Analysis of Higher and Lower PEEP in ARDS Patients: Systematic Review and Meta-Analysis

**DOI:** 10.1155/2022/5399416

**Published:** 2022-03-21

**Authors:** Min Liang, Xin Chen

**Affiliations:** ^1^Department of Intensive Care Unit, Sir Run Run Shaw Hospital, Affiliated to School of Medicine, Zhejiang University, Hangzhou, China; ^2^Department of Intensive Care Unit, Hangzhou Tumor Hospital, Affiliated to School of Medicine, Zhejiang University, Hangzhou, China

## Abstract

**Background:**

Positive end-expiratory pressure (PEEP) refers to the positive pressure in the respiratory tract at the end of the exhalation when we use a ventilator. The differences of higher PEEP and lower PEEP on clinical outcomes in acute respiratory distress syndrome (ARDS) patients are less well known.

**Methods:**

A comprehensive literature search of all randomized control trials (RCTs) was conducted using PubMed, Embase, World Health Organization (WHO) Global Index Medicus, WHO clinical trial registry, and Clinicaltrials.gov. Inclusion criteria included RCTs comparing the clinical outcomes of higher and lower PEEP in ARDS patients.

**Results:**

Eleven studies were included in the final analysis. In the higher PEEP group, the hospital mortality, 28-day mortality, and ICU mortality showed no significantly lower risk compared to the lower PEEP group (RR = 0.92, 95% CI 0.80–1.05, *p* = 0.22; RR = 0.88, 95% CI 0.73–1.05, *p* = 0.15; RR = 0.84, 95% CI 0.67–1.05, *p* = 0.12; respectively). High certainty could be obtained that there is no significant difference between the clinical outcomes of higher PEEP and lower PEEP in ARDS patients.

**Conclusions:**

There is no significant difference of the hospital mortality, 28-day mortality, and ICU mortality between higher and lower PEEP in ARDS patients.

## 1. Introduction

Acute respiratory distress syndrome (ARDS) is caused by intrapulmonary and/or extrapulmonary causes. It is a clinical syndrome characterized by refractory hypoxemia and has attracted much attention due to its high mortality [1]. The etiology of ARDS is various, and the pathogenesis of ARDS caused by different etiology is different. The clinical manifestations are acute onset, respiratory distress, and hypoxemia which is difficult to be corrected by conventional oxygen therapy. At present, “Berlin definition” is used to make diagnosis and stratification of severity of ARDS, and it is necessary to make differential diagnosis with many diseases [2].

Etiology of ARDS includes intrapulmonary cause and extrapulmonary cause [3]. Intrapulmonary causes include pneumonia, aspiration, pulmonary contusion, drowning, and inhalation of toxic substances. Extrapulmonary factors include severe systemic infection, severe multiple injuries (multiple fractures, flail chest, severe brain trauma, and burns), shock, high-risk surgery (cardiac surgery, major artery surgery, etc.), massive blood transfusion, drug poisoning, pancreatitis, and cardiopulmonary bypass. In addition, the etiology of ARDS can be divided into biological pathogenic agents and abiotic pathogenic agents. Biological pathogenic agents mainly include a variety of pathogens, such as bacteria, viruses, fungi, atypical pathogens, DAMPs, and malignant tumors. Abiotic pathogenic agents mainly include acid substances, drugs, toxic gas inhalation, and mechanical ventilation-related injury [4, 5].

At present, in addition to actively treating the primary disease, respiratory support technology is the main treatment method for ARDS, which aims to correct intractable hypoxemia, prevent alveolar collapse, reduce the degree of pulmonary edema, improve oxygenation, and relieve ventilator fatigue [6]. The treatment of ARDS includes mechanical ventilation and nonmechanical ventilation. Mechanical ventilation is the main treatment for ARDS patients. According to the different modes of mechanical ventilation, it can be divided into noninvasive ventilation and invasive ventilation [7]. Noninvasive ventilation relies on mask for ventilation, while invasive ventilation relies on endotracheal intubation or tracheotomy catheter for ventilation. The choice of the two depends on the specific condition and the timing [8, 9].

Positive end-expiratory pressure (PEEP) refers to the positive pressure in the respiratory tract at the end of the exhalation when we use a ventilator (usually positive pressure is applied only on the inhale and drops to zero on the exhalation). In this way, early alveolar closure can be avoided, and some alveoli that lose ventilation function due to exudation, atelectasis, and other reasons will expand so that the reduced functional residual volume will increase, and the purpose of improving blood oxygen can be achieved [10]. PEEP is similar to intermittent positive pressure respiration, but because of its longer duration of action, it has a wider range of effects on the respiratory and circulatory systems [11]. PEEP is the external pressure applied to the airway by the ventilator at the end of the patient's expiratory breath during mechanical ventilation. PEEP helps the lungs to expand and dilate collapsed alveoli. Acute lung injury reduces lung volume, lung compliance, ventilation/blood flow imbalance, and intrapulmonary shunt, leading to persistent hypoxemia and life-threatening complications. Appropriate PEEP is selected to reopen poorly ventilated alveoli, thereby improving lung compliance, ventilation/flow imbalance, and pulmonary shunt.

Many randomized controlled trials (RCTs) have compared the effect of higher PEEP and lower PEEP on reducing mortality in ARDS patients with inconsistent results [12–22], most likely due to variations in experiment design and methodological measurements. The differences of higher PEEP and lower PEEP on clinical outcomes in acute respiratory distress syndrome (ARDS) patients are less well known. Therefore, an explicit systematic review and meta-analysis were demanded to evaluate the difference of higher PEEP and lower PEEP on clinical outcomes in ARDS patients.

## 2. Materials and Methods

### 2.1. Study Selection

All RCTs to compare the effect of higher PEEP and lower PEEP on preventing mortality in ARDS patients were searched using PubMed (1966–2021), Embase (1980–2021), and World Health Organization (WHO) Global Index Medicus. Unpublished or ongoing studies were identified by checking clinical trials registers through Clinicaltrials.gov and WHO clinical trial registry. Literature in all languages was included in the search. Meta-analyses and systematic reviews were also hand-searched to find relevant literature that might have been missed by the initial search. The keywords used for search were “Positive end-expiratory pressure,” “acute respiratory distress syndrome,” “PEEP,” “ARDS,” “Mortality.” Furthermore, records from relevant searches were eventually hand-searched for further research. The asymmetry associated with the inclusion parameters of the published studies was finalized via discussion. The full set of published studies that were identified to be relevant for systematic review and meta-analysis were finalized according to the following set of inclusion parameters: (1) authentic research works, (2) documented in English language, (3) consisting of patients diagnosed with heart failure, and (4) includes details of patients taking medication for cardiovascular disease. As per the aim of the given study, prime attention was provided to the data where the patient cases related to heart failure were involved. There were multiple studies with the following category which were discarded: (1) insufficient data of the patients, (2) duplicity in published works, (3) nonclinical studies, (4) abstracts, conference papers, editorials, letters, or review studies, (5) research studies with no conclusions, and (6) insufficient patient data.

### 2.2. Data Extraction

Articles retrieved from the searches were evaluated independently by 2 reviewers using predefined standardized data extraction forms, and then, the data were evaluated by a third reviewer independently based on the US National Institute of Health National Heart, Lung, and Blood Institute (NHLBI) study quality assessment tool for controlled intervention studies [23]. Clinical outcome of interest was the hospital mortality, 28-day mortality, and ICU mortality as defined by the trial authors. The data pertaining to patients, the kinds of treatment, and methodology were abstracted (Table 1).

### 2.3. Meta-Analysis

The Preferred Reporting Items for Systematic Reviews and Meta-Analyses statement methodology [24] was adhered to. Relative risks (RRs) with a 95% CI for postoperative infectious complications of each trial were calculated to estimate treatment effects. Meta-analysis of the pooled data was performed using the fixed-effect model or random-effect model, depending on the heterogeneity of the included studies. If clinical heterogeneity was observed, data were analyzed using a random-effect model. Heterogeneity was quantified using the Cochrane's *Q* statistic and *I*^2^ statistic, with the values of 25%, 50%, and 75% signifying the limits of low, moderate, and high statistical heterogeneity, respectively [25]. A funnel plot was used to explore publication bias for the studies. All statistical analyses were performed using RevMan 5.4.

The risk of bias was evaluated using the Cochrane risk of bias tool. It was used to evaluate the selection bias, performance bias, detection bias, attrition bias, reporting bias, and other bias. The evidence quality was evaluated using the GRADEPro based on the results of systematic evaluation. To achieve transparency and implicity, the GRADE system classifies the certainty of evidence in one of four grades: high: further research is very unlikely to change our confidence in the estimate of effect; moderate: further research is likely to have an important impact on our confidence in the estimate of effect and may change the estimate; low: further research is very likely to have an important impact on our confidence in the estimate of effect and is likely to change the estimate; very low: any estimate of effect is very uncertain.

## 3. Results

### 3.1. Demographic Characteristics of the Studies

The literature search process, shown in Figure 1, identified 221 potential studies for full analyses. Eleven studies were finally included for further quantitative meta-analyses after exclusion [12–22] (Figure 1), involving a total of 3832 patients. Clinical outcome of interest was the hospital mortality, 28-day mortality, and ICU mortality. Of the 11 studies identified in the present analysis, 8 studies reported the hospital mortality, 8 studies reported the 28-day mortality, and 6 studies reported the ICU mortality. Only 4 studies included in the analysis reported all the three outcomes (Table 1).

### 3.2. Comparison of Hospital Mortality during Higher PEEP or Lower PEEP

Of the 11 studies identified in the present analysis, 8 studies reported the hospital mortality, including 3683 patients. Among these patients, higher PEEP was performed in 1827 patients, 766 patients died, and the hospital mortality was 41%, while lower PEEP was performed in 1856 patients, 805 patients died, and the hospital mortality was 43%. There was moderate heterogeneity between trials and it was significant (*I*^2^ = 55%, *p* = 0.03; Figure 2), so the random-effect model was applied. In the higher PEEP group, the hospital mortality showed no significant lower risk relative to the lower PEEP group (RR = 0.92, 95% CI 0.80–1.05, *p* = 0.22; Figure 2). In the funnel plot, all points are symmetrically distributed, indicating that there is no obvious publication bias (Figure 3).

### 3.3. Comparison of 28-Day Mortality during Higher PEEP or Lower PEEP

Of the 11 studies identified in the meta-analysis, 8 studies reported the 28-day mortality, including 3168 patients. Among these patients, higher PEEP was performed in 1567 patients, 576 patients died, and the hospital mortality was 37%, while lower PEEP was performed in 1601 patients, 610 patients died, and the hospital mortality was 38%. There was moderate heterogeneity between trials, and it was significant (*I*^2^ = 59%, *p* = 0.02; Figure 4), so the random-effects model was applied. In the higher PEEP group, the hospital mortality showed no significantly lower risk relative to the lower PEEP group (RR = 0.88, 95% CI 0.73–1.05, *p* = 0.15; Figure 4). In the funnel plot, all points are symmetrically distributed, indicating that there is no obvious publication bias (Figure 5).

### 3.4. Comparison of ICU Mortality during Higher PEEP or Lower PEEP

Of the 11 studies included in the final analysis, 6 studies reported the ICU mortality, including 2405 patients. Among these patients, higher PEEP was performed in 1186 patients, 514 patients died, and the hospital mortality was 43%, while lower PEEP was performed in 1219 patients, 549 patients died, and the hospital mortality was 45%. There was moderate heterogeneity between trials, and it was significant (*I*^2^ = 69%, *p* = 0.006; Figure 6), so the random-effects model was applied. In the higher PEEP group, the hospital mortality showed no significant lower risk relative to the lower PEEP group (RR = 0.84, 95% CI 0.67–1.05, *p* = 0.12; Figure 6). In the funnel plot, all points are symmetrically distributed, indicating that there is no obvious publication bias (Figure 7).

### 3.5. Publication Bias

Publication bias was assessed and visualized by using a funnel plot (Figure 5). A funnel plot is a simple scatter plot that reflects the estimated intervention effect of a single study with a given sample size or accuracy. The most common funnel plot is the estimated effect of each study on the horizontal axis and the sample size on the vertical axis. If there is bias, the funnel diagram will be asymmetrical and the bottom corner of the graph will be blank. In such cases, the effects calculated by meta-analysis may overestimate the efficacy of the intervention. The more pronounced the asymmetry, the more likely there is to be substantial bias. From Figures 3, 5, and 7, all points are symmetrically distributed, indicating that there is no obvious publication bias.

### 3.6. Risk of Bias Analysis

The risk of bias of the studies included is summarized in Figure 8. The selection bias, performance bias, detection bias, attrition bias, and other bias were evaluated by using the Cochrane risk of bias tool. Of the 11 studies, 2 had incomplete outcome data and 4 had selection reporting bias (18% and 36%, respectively). Attrition bias occurred during the study follow-up due to loss of follow-up, withdrawal, and no response. Use of appropriate statistical methods, such as intention-to-treat (ITT) analysis, can reduce this bias. Reporting bias occurs when research results are reported and can be avoided by registering research.

### 3.7. Evaluation of the Quality of Evidence

The GRADE system classifies the certainty of evidence in one of four grades: high, moderate, low, and very low.

The three clinical outcomes (hospital mortality, 28-day mortality, and ICU mortality) were all critical. High certainty could be obtained that there is no significant difference between the clinical outcomes of higher PEEP and lower PEEP in ARDS patients (Table 2).

## 4. Discussion

With the rapid increase of the ARDS incidence, the burden of ARDS diseases is gradually increasing. PEEP has been the common treatments for ARDS patients worldwide. It can be used in patients with spontaneous breathing through a face mask or endotracheal intubation. PEEP in this case is called continuous positive airway pressure. PEEP can also be used in conjunction with intermittent positive pressure mechanical ventilation to produce what is known as continuous positive pressure ventilation. The extent to which either form of PEEP may improve the oxygenation state depends on the degree to which the mean airway pressure increases. However, the difference between higher PEEP and lower PEEP was less known. In the present study, we evaluated the difference of them on clinical outcomes in ARDS patients systematically.

PEEP should be applied early in patients who have failed to respond to oxygen therapy. During mechanical ventilation, the inspiratory airway and alveoli are under positive pressure, and the airway and alveolar pressure are higher than atmospheric pressure when the airway opens at the end of expiratory. PEEP can improve the ventilation function of ARDS. Low levels of PEEP are often used in supine intubated patients [26]. Some researchers believe that low-pressure PEEP allows patients to maintain higher lung volume while breathing through a tracheal tube, thus helping to wean them off mechanical ventilation [27]. Hypoxemia in pulmonary diseases is mainly caused by intrapulmonary shunt, and adequate oxygenation is often not achieved even at FiO_2_ 1.0. When used at more than 5 cm H_2_O, PEEP generally improves PaO_2_ in these patients. PEEP also reduced FiO_2_ by 0.6 or less, thereby reducing the risk of oxygen poisoning [28].

Eleven studies were identified in the meta-analysis. In the higher PEEP group, the hospital mortality, 28-day mortality, and ICU mortality showed no significantly lower risk compared to the lower PEEP group. In all the funnel plots, all points are symmetrically distributed, indicating that there is no obvious publication bias. Attrition bias and reporting bias are the main two bias existed in the study. High certainty could be obtained that there is no significant difference between the clinical outcomes of higher PEEP and lower PEEP in ARDS patients. The complications of PEEP are related to lung volume and airway pressure. Air is pushed into the lungs at high pressure throughout the ventilation cycle to increase the volume of the lungs. Not only is air pumped into the lungs at high pressure during inhalation, it is more likely to cause barotrauma, or “volume injury,” but it is also more likely to reduce venous blood flow to the chest, lowering blood pressure and cardiac output.

There are some limitations should be acknowledged. First, there was significant clinical heterogeneity between studies. Therefore, the random-effects model was applied. Second, definitions of clinical outcomes were not specified among these studies, and differences in the definition of them can affect estimation of effect size. Third, differences in the treatment used between studies may account for heterogeneity, which may have influenced our results. Despite these limitations, the findings support higher PEEP is not different from lower PEEP when considering the incidence of clinical outcomes, including the hospital mortality, 28-day mortality, and ICU mortality as defined by each study. Further studies are required to be conducted to confirm the findings due to large clinical heterogeneity.

## Figures and Tables

**Figure 1:** PRISMA flow diagram showing the process of literature screening, study selection, and reasons for exclusion. PRISMA, preferred reporting items for systematic reviews and meta-analyses.

**Figure 2:** Forest plot of comparison of hospital mortality during higher PEEP or lower PEEP.

**Figure 3:** Funnel plot of included studies demonstrating the risk ratios of hospital mortality in the higher PEEP group compared to the lower PEEP group. SE indicates standard error.

**Figure 4:** Forest plot of comparison of 28-day mortality during higher PEEP or lower PEEP.

**Figure 5:** Funnel plot of included studies demonstrating the risk ratios of 28-day mortality in the higher PEEP group compared to the lower PEEP group. SE indicates standard error.

**Figure 6:** Forest plot of comparison of ICU mortality during higher PEEP or lower PEEP.

**Figure 7:** Funnel plot of included studies demonstrating the risk ratios of ICU mortality in the higher PEEP group compared to the lower PEEP group. SE indicates standard error.

**Figure 8:** Risk of bias analysis for the studies included.

**Table 1:** Characteristics of all randomized control trials comparing the effect of higher PEEP and lower PEEP on mortality (1966–2021).

Study name	No. of participants (high PEEP)	No. of participants (low PEEP)	Higher PEEP	Lower PEEP	Outcome of interest
Amato et al. [12]	29	24	Lower inflection point + 2 cm H_2_O	FiO_2_-PEEP	①②③
Ranieri et al. [13]	18	19	Lower inflection point + 2 cm H_2_O	FiO_2_-PEEP	②
Brower et al. [14]	276	273	FiO_2_-PEEP (ARDSnet)	FiO_2_-PEEP	①
Villar et al. [15]	50	45	Lower inflection point + 2 cm H_2_O	FiO_2_-PEEP	①③
Meade et al. [16]	475	508	FiO_2_-PEEP	FiO_2_-PEEP	①②③
Mercat et al. [17]	385	382	P_plat_	FiO_2_-PEEP	①②
Talmor et al. [18]	30	31	Transpulmonary pressure	FiO_2_-PEEP	②
Huh et al. [19]	30	27	Saturation decrease more	FiO_2_-PEEP	②③
Hodgson et al. [20]	10	10	PFiO_2_-PEEP	FiO_2_-PEEP	①
Kacmarek et al. [21]	99	101	PEEP + 35–45 cm H_2_O	FiO_2_-PEEP	①②③
Cavalcanti et al. [22]	501	509	PEEP + 2 cm H_2_O	FiO_2_-PEEP	① ②③

①: hospital mortality; ②: 28-day mortality; ③: ICU mortality.

**Table 2:** Higher PEEP compared lower PEEP in ARDS patients with different clinical outcomes of interest.

Certainty assessment							No. of patients		Effect		Certainty	Importance
No. of studies	Study design	Risk of bias	Inconsistency	Indirectness	Imprecision	Other considerations	Higher PEEP	Lower PEEP	Relative (95% CI)	Absolute (95% CI)		
*Hospital mortality*												
8	Randomized trials	Not serious	Not serious	Not serious	Not serious	Strong association	766/1827 (41.9%)	805/1856 (43.4%)	RR 0.97 (0.89 to 1.04)	13 fewer per 1,000 (from 48 fewer to 17 more)	High	Critical

*28-day mortality*												
8	Randomized trials	Not serious	Not serious	Not serious	Not serious	None	576/1567 (36.8%)	610/1601 (38.1%)	RR 0.96 (0.88 to 1.05)	15 fewer per 1,000 (from 46 fewer to 19 more)	High	Critical

*ICU mortality*												
6	Randomized trials	Not serious	Not serious	Not serious	Not serious	None	514/1186 (43.3%)	549/1219 (45.0%)	RR 0.96 (0.88 to 1.04)	18 fewer per 1,000 (from 54 fewer to 18 more)	High	Critical

CI: confidence interval; RR: risk ratio.

## Data Availability

The data used to support this study are available from the corresponding author upon request.
